This article has been retracted.

# Beyond the Psychopathological Approach to Study the Relationship between Body Dissatisfaction and Suicide: A Moderate and Mediated Analysis

**DOI:** 10.1155/2022/6285473

**Published:** 2022-10-13

**Authors:** Wei Jiang

**Affiliations:** Faculty of Education, Huaibei Normal University, Huaibei 235000, China

## Abstract

This paper provides a comprehensive review of the literature to date on body dissatisfaction and suicide. A moderate and mediated regression analysis suggests that the relationship between these two variables is mediated by depression, anxiety, impulse control, self-esteem, and hopelessness. The relationship is not moderated by gender, ethnicity, or socioeconomic status. The implications for mental health practitioners are discussed in relation to management strategies for body dissatisfaction and suicide risk. Another finding showed that psychological distress had a significant effect on performance achievement and served as a mediating variable for the effect of social justice on performance achievement. This study only focused on the effect of psychological distress on the performance achievement of human resources in the context of Islamic microfinance institutions. Besides, in explaining the model, this study only focused on one point of view of the grand theory, i.e., social exchange theory. This study provided information on alternative strategies in managing and minimizing the risks of psychological distress to improve performance achievement in Islamic microfinance institutions. Apart from that, this study also provided an overview of how to manage social exchange relationships in the context of an organization, so they could be well-maintained. This study examined the effect of psychological distress on the performance achievement of human resources in the context of Islamic microfinance institutions. This study also specifically examined the role of formal justice and social justice as an antecedent of psychological distress. Eventually, this study used the perspective of social exchange theory for the first time in explaining the psychological distress model on the performance achievement of human resources.

## 1. Introduction

The hazards of psychological discomfort are one of the significant challenges that practitioners and scholars in the field of human resource management should pay attention to in the industrial revolution period. If the work environment is unpredictable and demands the capacity to adapt, all members of the company may experience psychological suffering. This situation necessitates that all members of the organization use their skills to their full potential, yet this can lead to psychological discomfort if the goals are not met. Instead of being able to make a good contribution, stress can lead to a decline in mental health, resulting in poor performance. This condition is consistent with experts' observations that psychological discomfort has a detrimental impact on employee and organizational performance [1].

Other organizational elements can also cause psychological pain; in the context of social exchange theory, the organization is referred to as an arena of exchange that includes leaders and members of the organization [2]. There is a view that disputes arise often in trading processes, resulting in psychological suffering. In most cases, conflicts arise because of unfair trade practices [3]. In the context of an organization, inequity is linked to issues of formal and social justice. Employees believe they are unappreciated because of such unfairness and that their efforts for the leadership and the company are in vain. Employees that are emotionally susceptible typically experience psychological suffering, even mental health worsening, when this situation is not acceptable [4, 5]. Employees suffering from significant psychological anguish lose attention at work, resulting in lower production quality and quantity than under normal circumstances. To put it another way, this condition implies that psychological anguish may contribute to poor performance.

This research contributed to the science and practice of human resource management in various ways. To begin, we looked at how psychological discomfort influences human resource performance in a business. In practice, psychological anguish leads organizational members to lose concentration, making it impossible for them to make their best contributions, resulting in a drop in performance [6, 7]. We think that reducing the risk of psychological discomfort can lead to improved performance.

Second, we applied the perspective of social exchange theory to understand the impact of psychological discomfort on human resource performance. Exchanging goods and services can frequently lead to disappointment and discontent among all parties concerned [8]. This illness is unmistakably the result of a bad emotional reaction. Injustice is one of the variables that are thought to produce unpleasant emotional responses throughout the trading process [9]. Our opinion that social exchange theory is important to explaining psychological suffering has been bolstered by referring to this remark. Furthermore, few researches look at psychological suffering via the lens of social exchange theory.

Finally, we looked at how organizational characteristics contribute to psychological suffering. Psychological distress, according to specialists, is an emotional condition that an individual experiences as a response to a specific stress or request that results in losses and unmet demands [10]. Requests that result in losses in the framework of an organization, in our judgement, amount to both formal and social wrong. Inequity in the workplace and in society is a strong predictor of psychological suffering [11, 12]. Because a presumption arises that not all of their efforts are acknowledged and that their presence is neglected, injustice produces a negative emotional response in an individual. Excessive negative emotional responses might lead to serious psychological suffering in a person [13, 14]. As specialists have pointed out, injustice has an impact on psychological discomfort [15]. Unfortunately, little research has been done on the effects of formal and social justice on psychological discomfort, particularly in the realm of organizational justice.

Finally, in the context of Islamic microfinance firms in Indonesia, we investigated the impact of psychological distress on employee performance. There are few empirical researches on the impact of psychological strain on performance, particularly in Islamic microfinance organizations. This is due to the belief that financial institutions face greater labor pressure than nonfinancial institutions [16], as well as a significant risk of organizational unfairness, particularly in microfinance firms.

## 2. Literature Review

### 2.1. Social Exchange Theory

According to [17], social exchange is an exchange of both material and/or nonmaterial goods that involves no less than two parties. Another definition of social exchange refers to voluntary actions of an individual who is motivated by returns that they expect to receive and that they usually obtain from others [18]. In addition, Emerson [19–22] assumed that social exchange is a resource that will continue to exist if there is a return in value that is of equity. The perspective of social exchange theory describes an organization as an arena of exchange that involves leaders and employees. In general, a person decides to become a member of an organization because s/he has an expectation to obtain benefits. In reality, the exchange relationships do not always go as expected by the parties involved; there are risks of negative affective conditions due to a conflict during the exchange. This conflict can be triggered by injustice perceived by one of the parties. Injustice encourages the aggrieved party to respond to the injustice as a protest for their anger and disappointment by deliberately lowering the quality and quantity of inputs or outputs. A number of experts reveal that low levels of justice trigger higher negative emotional reactions [13, 23]. Negative emotional reactions can be displayed through a variety of destructive behaviours, including anger, anxiety, and distress [24], eventually leading to a reduced performance [25].

### 2.2. Formal Justice

Formal (procedural) justice represents the fairness of the procedure for determining outcomes [26]. Intellectual and emotional recognition will be formed from procedural justice, which then creates trust and commitment that build voluntary cooperation in the implementation of strategies [27]. Dharmawati et al. [28] explained that formal (procedural) justice is responsible for a decrease in performance. This statement is in line with a number of studies, showing that formal justice has a significant effect on employee performance [29, 30]. Under different conditions, procedural injustice could trigger intellectual and emotional anger as well as distrust and hatred [31–33]. This condition is very likely to occur, particularly in relation to exchange relationships. Procedural injustice could also trigger a perception that the inputs contributed by one party are meaningless for the other party involved in the exchange. This certainly causes disappointment and anger that may lead to psychological distress. This assumption is in line with the findings of previous empirical studies, showing that formal justice has a significant effect on psychological pressure [11, 15]. Based on the empirical findings and assumptions that have been built, alternative hypotheses are proposed as follows:

*H*_1_: formal justice has a positive effect on employee performance.

*H*_2_: formal justice has a negative effect on psychological distress.

### 2.3. Social Justice

Social justice in the context of an organization is represented as the communication perceived by employees and how the management treats them [34]. A study revealed that social or interactional factors have a significant effect on motivation and lead to increased work outcomes [34]. Pakpahan et al. [35] in a study of employees of PT Telkomsel Indonesia in the East Java region found that the interactional justice dimension had a significant effect on employee performance. This is in line with the findings of other studies, showing that social justice can affect performance [30, 36, 37]. The perception of unfulfilled social justice in the form of the leaders not behaving politely, not respecting employees, and sharing information inappropriately can trigger the aggrieved party to have negative affective conditions. Lucas found that social justice can affect mental health and negative emotional conditions such as depression. This finding is in accordance with a number of previous studies and strengthens the assumption that justice can serve as a significant antecedent of psychological distress [12, 15]. Based on the empirical findings and assumptions that have been built, alternative hypotheses are proposed as follows:

*H*_3_: social justice has a positive effect on employee performance.

*H*_4_: social justice has a positive effect on psychological distress.

### 2.4. Psychological Distress

In general, a negative affective condition occurs because exchange relationships do not run well. This condition can be manifested in the form of expressions of regret, disappointment, and anger. A negative affective condition can be experienced by all parties without exception, and, when not properly handled, this condition may result in psychological distress and mental health deterioration. According to Robert and Hockey [38], there is a decrease in individual motivation and efforts when experiencing psychological distress. In addition, psychological distress may make individuals unable to manage their roles optimally, thus decreasing their work achievement. Lim and Tai [25] in a study of employees of nonprofit organizations in Singapore found a significant negative effect of psychological distress on work performance. Hilton et al. [17, 39, 40] found that moderate and high levels of psychological distress had a significant correlation with a decrease in the success at work. This is similar to the findings of a recent study that psychological distress had a significant effect on individual performance [1, 6, 7]. Based on the empirical findings and the assumptions that have been built, alternative hypotheses are proposed as follows:

*H*_5_: psychological distress has a negative effect on employee performance.

### 2.5. Mediation Effect of Psychological Distress

According to [3] in the perspective of social exchange theory, an organization reflects an arena of exchanges, where the decision taken by someone to join as a member of the organization is due to an expectation to gain benefits. Exchange relationships basically should consider the aspect of balance in relation to the input and output contributions of each of the parties involved in the exchange [2]. The risk of conflicts could lead to a decrease in the quality of the exchange relationships due to an imbalance between input and output contributions. This imbalance is a representation of injustice which then triggers a negative emotional response from the aggrieved party. Such negative emotional response, if uncontrolled, may cause psychological distress and mental health deterioration. When this condition cannot be overcome, employees may lose their focus at the workplace. As a consequence, the quality and quantity of work are not optimal. Referring to this assumption, alternative hypotheses are proposed as follows:

*H*_6_: psychological distress mediates the effect of formal justice on employee performance.

*H*_7_: psychological distress mediates the effect of social justice on employee performance (see Figure 1).

## 3. Research Methods

### 3.1. Data Collection and Analysis

This study involved 194 managers and employees of Islamic Microfinance Institutions in the Special Region of Yogyakarta, Indonesia. The data were collected by a survey using the convenience sampling method. The survey was conducted using a questionnaire referring to the six-point Likert scale. For the hypothesis testing and data analysis, this study used a structural equation modelling (SEM) approach with the analysis moment structure (AMOS) software version 24.00.

### 3.2. Measurement Variables

Psychological distress in this context was measured by six indicators developed by [41]. Meanwhile, employee performance was measured by five indicators from the dimensions of in-role performance by referring to [42]. Finally, in their roles as exogenous constructs, formal justice (procedural justice) and social justice (interactional justice) were measured by referring to the indicators developed by Colquitt and Tjahjono [43, 44].

## 4. Results

### 4.1. Measurement Model

The first-order confirmatory factor analysis (CFA) showed that there was one indicator variable with a loading factor < 0.5, namely the formal justice construct “I can file appeal or protest the (results) achieved by the procedure (FJ6)”; the item should be removed to obtain an indicator variable with better validity. The first-order confirmatory factor analysis (CFA) also showed the goodness of fit value of the employee performance construct and found six indices with good fit criteria (RMR, RMSEA, GFI, AGFI, TLI, and GFI). In the formal justice construct, there was only one index with good fit criteria (RMR), and two of them fell in the marginal fit category (GFI and CFI). In the social justice construct, no index was found to have good fit criteria. For the psychological distress construct, only three indices were found to have good fit criteria (GFI, TLI, and CFI) and one of them fell in the marginal fit category (AGFI). According to Hair et al. [21], it requires at least three or four indices with good fit criteria in order for the model to be considered appropriate. Based on this opinion, it is necessary to revise and modify several constructs (formal justice and social justice) to obtain a more appropriate model, as shown in Tables 1–3.

### 4.2. Structural Model

The revised structural model showed that the overall loading factor of all the indicators was >0.5, meaning that all the construct indicators were valid. The revised structural model also showed that the overall convergent validity of the constructs was VE > 0.5, AVE > 0.5, and CR > 0.7, meaning that the construct items after the model was revised were reliable. The AVE square root of each latent construct was higher than the correlation value between the constructs, meaning that each construct met the discriminant validity assumption. Finally, the revised structural model found five indices with good fit criteria (RMR, RMSEA, CMIN/DF, TLI, and CFI), so the structural model was considered appropriate (see Figure 2).

Univariate data normality showed that most of the critical ratio (CR) on skewness was greater than ±2.58. Meanwhile, the multivariate data normality showed that the critical ratio (CR) in kurtosis was 25.552 or greater than ±2.58. Nonetheless, some experts argue that the multivariate normality assumptions can also be met with a critical kurtosis not greater than 30 [45, 46]. Furthermore, the Mahalanobis distance showed no data exceeding 54.052, meaning that there were no multivariate outliers. Finally, the correlation between the independent variables was 0.589 < 0.85, indicating no multicollinearity in the model (see Table 4).

The hypothesis testing in Table 5 shows that the standardized regression coefficient of the formal justice construct on employee performance was 0.347 with a CR of 3.349 > 1.96, meaning that the first hypothesis was accepted. The standardized regression coefficient of the social justice construct on employee performance was 0.040 with a CR of 0.445 < 1.96, indicating that the second hypothesis was rejected. The standardized regression coefficient of the formal justice construct on psychological distress was -0.243 with a C.R of −2.384 > 1.96, meaning that the third hypothesis was accepted. The standardized regression coefficient of the social justice construct on psychological distress was -0.351 with a C.R of −3.499 > 1.96, indicating that the fourth hypothesis was accepted. The standardized regression coefficient of the psychological distress construct on employee performance was -0.283 with a CR of −3.223 > 1.96, meaning that the fifth hypothesis was accepted.

### 4.3. Mediation Effect

The results of the direct effect and indirect effect test in Table 6 show that the value of the direct effect of the formal justice construct on employee performance through psychological distress was 0.347, greater than the indirect effect of the formal justice construct on employee performance through psychological distress (0.069). This means that psychological distress did not mediate the effect of formal justice on employee performance, so the sixth hypothesis was rejected. Meanwhile, the value of the direct effect of the social justice construct on employee performance through psychological distress was 0.040, lower than the indirect effect of the social justice construct on employee performance through psychological distress (0.099). This means that psychological distress mediated the effect of social justice on employee performance, so the seventh hypothesis was accepted.

## 5. Discussion

The finding of this study proved that formal justice had a significant effect on employee performance achievement and this is in line with the finding of several previous studies [28–30]. The fulfillment of formal justice encourages employees to contribute positively, manifested in the form of optimal efforts to develop the organization. Employees perceive that the fulfillment of formal justice is a concrete proof of the organization's commitment to paying attention and being responsible for its members. Another finding of this study proved that both formal justice and social justice also had a significant effect on psychological distress and this is in line with the findings of several experts in relevant previous studies [11, 12]. Nonfulfillment of formal and/or social justice can trigger a negative emotional response in the form of disappointment which can cause psychological distress. The perception of injustice can create a negative stigma, i.e., that the leader or organization neither appreciates the efforts made by its members nor pays attention to the welfare of the members. When employees are unable to accept these conditions, they might have to experience negative affective conditions which lead to psychological distress [15].

The next finding showed that psychological distress had a significant effect on employee performance. This is in accordance with the statement of experts in several relevant previous studies [1, 6, 7]. Employees revealed that psychological distress they experienced from work or unfair treatment of their leaders could make them lose focus at the workplace, consequently leading to a decreased quality and quantity. This condition should be overcome properly and immediately, unless it will have a significant effect in the form of losses. Furthermore, this study proved that psychological distress mediated the effect of social justice on employee performance achievement. The nonfulfillment of social justice reflects that leaders are disrespectful to the members, eventually triggering distrust among employees to their leaders [47]. When leaders treat their employees unfairly, it will also create a negative stigma that these leaders neither care nor appreciate the existence of the members in the organization. Emotionally vulnerable employees will get angry, disappointed, and not accepting; when this condition remains, this may lead to severe psychological distress [48]. Uncontrolled psychological distress causes a person to lose focus at the workplace, making them unable to contribute optimally to the organization, thus decreasing the performance.

Finally, this study found that social exchange theory was relevant to explaining the role of psychological distress as a mediating variable for the effect of social justice on employee performance. In exchange relationships, conflicts between the parties involved are common. These conflicts may occur due to injustice committed or received by each of the parties [49]. Therefore, it is believed that exchange relationships are at risk of triggering negative emotional state. The parties who are unable to control their emotions could experience psychological distress or even mental health deterioration [4]. When this condition persists and cannot be properly managed, it can disrupt the quality of the exchange relationships, so the goal of the exchange relationships cannot be achieved optimally.

## 6. Conclusion and Implications

This study has proven that psychological distress has a significant effect on performance achievement. There will be positive benefits when psychological distress can be managed. On the other hand, there will be negative effects when psychological distress is not well managed. The findings of this study support the findings of several previous studies that psychological distress has a negative effect on performance achievement. This study also confirms the relevance of the social exchange theory in explaining psychological distress. Exchange relationships are inseparable from conflicts, mainly because there is an unfair party in terms of contributions, which in turn triggers disappointment, leading to psychological distress. Such injustice can be in the terms of formal (procedural) justice and social justice related to the behaviour of superiors to subordinates. Perceived injustice creates a perception among employees that they are not appreciated, then they will respond to it in the form of protest, one of which is by intentionally reducing their input or output contributions. On the other hand, the presence of justice can lower the risk of employees experiencing psychological distress. Justice helps employee have a perception that they are valued, recognized, and needed, and their superiors and the organization are committed and responsible for them. This then encourages the employees to make optimal contributions for the leadership and organization.

The findings of the study on the consequences of psychological distress can serve as a precaution to start realizing the risks of psychological distress. This study can also be used as a strategic alternative in managing the risks of psychological distress to achieve more optimal performance. In addition, these findings can also serve as an effective strategy to minimize conflicts that could be found in exchange relationships, allowing for the objective of the exchange to be more effectively achieved, namely to provide fair benefits for all the parties involved in the exchange. Finally, the findings can be used as the first step to start developing and conducting an in-depth and comprehensive study on the risk of psychological distress in various business sectors and in an organization.

## Figures and Tables

**Figure 1:** SEQ Figure \^∗^ Arabic 1 empirical model.

**Figure 2:** Structural model revised.

**Table 1:** Result of confirmatory factor analysis (CFA).

Construct	Items	Loading factor	VE	AVE	CR
Psychological distress	PD1	0.716	0.613	0.782	0.874
	PD2	0.655			
	PD3	0.596			
	PD4	0.870			
	PD5	0.807			
	PD6	0.730			

Formal justice	FJ1	0.675	0.518	0.720	0.827
	FJ2	0.651			
	FJ3	0.707			
	FJ4	0.651			
	FJ5	0.701			
	FJ6	0.398			
	FJ7	0.650			

Social justice	SJ1	0.904	0.616	0.785	0.913
	SJ2	0.917			
	SJ3	0.936			
	SJ4	0.607			
	SJ5	0.632			
	SJ6	0.609			
	SJ7	0.623			
	SJ8	0.624			
	SJ9	0.686			

Employee performance	EP1	0.735	0.747	0.873	0.926
	EP2	0.864			
	EP3	0.921			
	EP4	0.893			
	EP5	0.802			

**Table 2:** Measurement of structural model revised.

Model	*X* ^2^	DF	*P*	RMR	RMSEA	GFI	AGFI	CMIN/DF	TLI	CFI
Goodness of fit indices for measurement model revised										
Model revised	566.77	279	0.00	0.048	0.073	0.833	0.790	2,031	0.905	0.918

**Table 3:** Continuation of Table 2.

Construct	Items	Loading factor	VE	AVE	CR
Psychological distress	PD6	0.635	0.613	0.782	0.874
	PD5	0.693			
	PD4	0.626			
	PD3	0.811			
	PD2	0.823			
	PD1	0.780			

Formal justice	FJ7	0.615	0.518	0.720	0.827
	FJ5	0.595			
	FJ4	0.651			
	FJ3	0.742			
	FJ2	0.612			
	FJ1	0.705			

Social justice	SJ9	0.633	0.616	0.785	0.913
	SJ8	0.552			
	SJ7	0.561			
	SJ6	0.539			
	SJ5	0.600			
	SJ4	0.567			
	SJ3	0.955			
	SJ2	0.935			
	SJ1	0.913			

Employee performance	EP1	0.805	0.747	0.873	0.926
	EP2	0.893			
	EP3	0.916			
	EP4	0.867			
	EP5	0.734			

**Table 4:** Discriminant validity.

Construct	FJ	SJ	PD	EP
FJ	0.720			
SJ	0.353	0.785		
PD	0.182	0.248	0.782	
EP	0.263	0.162	0.199	0.873

**Table 5:** Hypotheses test.

		Estimate	SE	CR	*P*	Remark
PD	FJ	-0.243	0.201	-2.384	0.017	Significant
PD	SJ	-0.351	0.160	-3.499	^∗∗∗^	Significant
EP	PD	-0.283	0.056	-3.223	0.001	Significant
EP	FJ	0.347	0.130	3.349	^∗∗∗^	Significant
EP	SJ	0.040	0.092	0.445	0.657	Not significant

**Table 6:** Direct and indirect effect.

	SJ	FJ	PD	EP
Standardized direct effect				
PD	-0.351	-0.243	0.000	0.000
EP	0.139	0.415	-0.283	0.000

Standardized indirect effect				
PD	-0.351	-0.243	0.000	0.000
EP	0.040	0.347	-0.283	0.000

## Data Availability

The data used to support the findings of this study are included within the article.
